The article "An ethnobotanical study of wetland flora of Head Maralla Punjab Pakistan" was retracted in 2023. Reasons: a conflict of interest; concerns about the peer review; concerns about the authorship.

# An ethnobotanical study of wetland flora of Head Maralla Punjab Pakistan

**DOI:** 10.1371/journal.pone.0258167

**Published:** 2021-10-14

**Authors:** Muhammad Sajjad Iqbal, Khawaja Shafique Ahmad, Muhammad Azhar Ali, Muhammad Akbar, Ansar Mehmood, Fahim Nawaz, Syed Atiq Hussain, Noshia Arshad, Saba Munir, Hamna Arshad, Khizra Shahbaz, Rainer W. Bussmann

**Affiliations:** 1 Department of Botany, University of Gujrat, Gujrat, Pakistan; 2 Department of Botany, University of Poonch Rawalakot, Azad Jammu & Kashmir, Pakistan; 3 Institute of Crop Science (340h), University of Hohenheim, Stuttgart, Germany; 4 Department of Agronomy, MNS, University of Agriculture, Multan, Pakistan; 5 Department of Ethnobotany, Institute of Botany, Ilia State University, La Paz, Bolivia; Mirpur University of Science and Technology, PAKISTAN

## Abstract

**Background:**

Wetlands are biologically diverse and highly productive ecosystems that support one-third of all threatened and endangered plants of the world. Wetland plants have been studied ethnobotanically much less than terrestrial plants, including in Pakistan, thus information about the uses of local wetland plants in traditional healthcare system is scare. Head Maralla is a non-recognized wetland with diversified flora that has been focused of the current study.

**Methods:**

The ethnobotanical data were collected from four sites viz., River Tavi, Upstream Chenab, River Manawarwala Tavi, and Bhalolpur through questionnaire and interviews during field trips. Quantitative indices including informant consensus factor (ICF), cultural significant indext (CSI), relative frequency of citation (RFC), and use value (UV) were used to analyze the data.

**Results:**

On the whole, 119 plant species were identified belonging to 54 families, of which 87 species were dicot, 12 monocots, 11 aquatic, 5 ferns, and 4 species were bryophytes. Of these, 50% of the plant species were utilized for therapeutic purposes, followed by leaves which had more than 20% usage of total consumption. Herbs were the primary source of medicine (73 spp) followed by trees (22 spp), weeds (11 spp), shrubs (9 spp), foliose (2 spp) and thaloids (2 spp) in the area. F_ic_ ranged from 0.66 to 0.93 for constipation and respiratory disorders with an average F_ic_ of 0.87 reflecting a high consensus among the informants about the use of plants to treat particular ailment. Major ailments viz., urination (14%), cough (8.40%), cold (6.70%), stomach (5.90%), asthma (5.90%), skin infection (5%), constipation (5%), and diarrhea (4%) etc., were treated with local plant recipes. The highest CSI value was found for *A*. *vesica* (7.55) widely used in respiratory disorders and in digestive problems. RFC ranged from 0.92 to 0.15 with the maximum value obtained for *R*. *communis* (0.95). The use values ranged from 0.03 to 0.90 with the maximum use value for *R*. *communis* (0.90). A positive correlation was found between CSI and RFC (r = 0.29), and CSI and UV (r = 0.29). The JI values ranged from 7.14 to 0.14 indicating strong affinity with Samahani valley, Azad Kashmir, Pakistan. Unique species *Osmunda regalis* was first time reported from Pakistan with novel uses for renal and blood purifier. Fifteen percent (15%) plants contribute as fodder species consumed by local community for livestock while almost 6.7% species were utilized for timber and fuel purposes.

**Conclusion:**

The ecosystem of Head Maralla provide a complex habitat for aqauatic, terrestrial, and agriculture wetland vegetation. It is suggested that conservation efforts should be made to conserve the ethnoecological knowledge of these areas and pharmacological studies should be conducted for noval drug synthesis in future.

## Introduction

Wetland in contrast to terrestrial ecosystems, have received little ethnobotanical attention, despite the fact that wild wetland plants play a significant role in the daily lives of people who live in and around wetlands [1, 2]. Plants are collected from wetlands for a number of reasons, including medicine, food, and building materials, as well as to sell for profit [3–5]. Wetlands are particularly vulnerable to loss or deterioration due to urbanization [6, 7], which can alter their area and species composition, resulting in large biodiversity loss [8]. Wetlands have progressively been lost and degraded due to human activities [9], and some concrete attempts are needed to restore the degraded wetlands [10].

From 1996 to the present, ethnobotanical reports on traditional knowledge legacy have been reported in Pakistan [11–14]. According to literature, the Himalayan mountains are home for 70% of wild plants and animals, which meet 70–80% of human demands for traditional medicines and healthcare [15, 16]. Head Maralla is most likely located in the Himalayan foothills as a wildlife hotspot. Ethnobotanical information is a treasure that is not just found in rural regions, but also in metropolitan areas since it is safer, less expensive, and has fewer negative effects [17]. About 400 plant species are utilised widely in traditional remedies, according to the National Institute of Health (NIH) and around 900 single medicines and 500 compound formulations are recognised in Pakistan’s Tibbi Pharmacopoeia [18]. Twenty-seven indigenous herbal companies have been approved for commercial production, and their revenue is equivalent to that of international corporations in Pakistan. Several Hakim Khanas exist around the country that are not properly registered with a recognised agency [19].

Furthermore, Pakistan’s northern and northwestern regions include a wide range of plant species [20]. Pakistan is believed to have 400–600 medicinal plants out of a total of 5700 [21]. Local people utilise herbs such as isphaghol, sweet fennel, black cumin, black seeds, bishops’ weed, milk thistle, Indian hemp, Datura, Sassurea, and Trianthma sp. Plant components such as rhizome, fruits, leaves, root, and bark are commonly used to cure cough, asthma, cold, pneumonia, hepatitis, kidney stones, anti-malaria, smallpox, heart, and sexual problems, among other ailments, thus plants hold great wealth for a healthy living [22, 23].

Traditional plant knowledge has long played an essential part in people’s lives, and it has the potential to play role in future for the long-term sustainability of communities and economies [24]. Among the plant diversity, 300 species are utilised as natural colours and flavouring agents not only in the culinary, pharmaceutical, cosmetics, and perfume industries, but also in traditional healthcare. Because to its climate and topography, Pakistan has a unique biodiversity [25–27]. Targets must be set in order to address future health issues. Plant product development has necessitated ethnobotanical evaluation via natural plant resource conservation and preservation [20, 28].

Twenty species out of a total of 20,000 provide 90% of all food [21]. Consequently, global heritage is required to be preserved for future generations, as it ensures a region’s socioeconomic activities by preserving traditional knowledge across areas [29]. The uses of plants and their products especially herbal medicines are not only evident from developing countries but also in developed countries in Europe and North America, where market sector is increasing at a rate of 10–20 percent per year [30].

The Head Maralla is floristically highly rich. The area has never been explored for ethnobotanical research. The climate in the region is quite variable. By occupation, the farmer community dominates, while government personnel come in second. Young people with poor literacy levels are eager to serve in foreign nations in order to benefit from higher living standards. The majority of women are housewives, with only a small percentage working in government. Both men and women are engaged (self-employed) in collection and trade of wild plants Plants are mostly utilised for food, shelter, and medicinal substances, with the bulk of the material being discarded. Scientific information regarding the usable portions, cultural practises, management, harvesting, timing of collection, processing, and packing are all insufficient, resulting in post-harvest losses on the one hand and a drop in national revenue on the other. Because indigenous knowledge is diminishing, this study was designed with the primary goal of quantifying the ethno-medicinal value of plants of the Head Maralla in the Punjabi districts of Sialkot and Gujrat, preserve the valuable folk knowledge about medicinal plants, and share the information with other communities through published literature.

## Material and methods

### Ethics statement

The study was approved by the Institutional Ethics Committee through No. UOG/ASRB/Botany/02/7881. Verbal informed consent was obtained from each informant before conducting the interview process.

### Study area

Head Maralla is situated at the foothills of Himalaya and lies between longitude 32°39’55.9 North and latitude 74°27’54.4 East at elevation of 233 m a.s.l. (Fig 1). The Chenab River’s primary water controlling structure, the headwork, was built in 1968. Fig 1 depicts a map of several locations. GPS (Global Positioning System) was used to choose and create the map. River Tavi (RT), Upstream Chenab (UC), River Manawarwala Tavi (RMT), and Bhalolpur side (BLP) were chosen as the sites for plant collection and observations (Fig 2). The temperature in the area is hot and humid, and the sites are riverine, with a lot of wetlands. The soil in the region is primarily sandy, with some loamy areas. These three rivers, Chenab, Tavi, and Manawarwala, flood the area during the monsoon season (Fig 2)

**Fig 1:** Map of Head Maralla showing four respective sites of the study area.

**Fig 2:** Pictorial view of four sites of the study area are showing near the Head Maralla.

#### Demographic information

The study region is located between two of the country’s most industrially significant cities, Sialkot and Gujrat. Sialkot is located in the Punjab province’s north-east corner. It is Pakistan’s 12th most populated city and is known for its entrepreneurial culture and economic climate, according to "The Economist." Surgical equipment, sports, musical instrumentation, and cutlery accounted for roughly $2.5 billion in 2019, accounting for nearly 10% of Pakistan’s total exports contribution [31]. During the Indus Valley civilisation, Sialkot was an agricultural region with woods, and it was also known as the winter capital of the State of Kashmir.

Sialkot District has a long history that dates back thousands of years. Since its inception, it has passed through the hands of Aryans, Persians, Greeks, Hindus, Buddhists, Muslims, Sikhs, and British rulers until becoming the modern-day federation of Pakistan. The district of Sialkot covers a total size of 3,016 square kilometres [32]. According to unpublished statistics from the 6th population and housing census 2017, the district had a population of almost 4.7 million people, compared to 595,000 according to Demographia World Urban Areas Annual Edition [32]. Urbanization accounted for around 35% of the population. Gujrat is a historic city situated between the Jhelum and Chenab rivers. It is located between Mirpur (northeast) and Jhelum (northwest), and it divides Jhelum district from it. River Chenab flows on the east side, southeast, dividing it from Gujranwala and Sialkot, while Mandi Bahauddin is located on the west. It is administratively divided into four tehsils Kharian, Jalal Pur Jattan, Sarai Alamgir, and Gujrat itself. Gujrat District covers a total size of 3,192 square kilometres. According to unpublished statistics from the 6th population and housing census 2017, the total population of Gujrat district is over 3.1 million. Moreover 37% of the ladies in the urban population were female. Punjabi is the district’s most common language, spoken by 98 percent of the population according to the 1998 census, with Urdu accounting for 1.1 percent [33].

#### Climate and ecology of study area

According to the topography and climate of the area, summers are hot and humid, while winters are cold,. The warmest months are May, June, and July. During the winter, minimum temperatures have been as low as -2°C, with maximum temperatures ranging from 40 to 50°C. The region is primarily agricultural, having plain and rich terrain. Monsoon season is the beauty of the area (mid-July to mid-August), when the weather is scorching during the day and cools down significantly at night. These days have a low humidity level. Mild to moderate weather may be found during the winter months, from mid-November to March, with significant rains on occasion. The yearly rainfall averages 1000 mm [11–13]. The climate in this district is moderate, with hot summers and chilly winters. The daytime temperature can reach up to 50°C during the summer, but the hot spells are comparatively shorter due to proximity of Azad Kashmir Mountains. The winter months are mild with temperatures seldom dropping below 2°C. The average rainfall in the Kashmir border is above 1000 mm, 750 mm in Kharian, 670 mm in Gujrat, and 500 mm in Dinga.

#### Data of agricultural land

According to the Agriculture Department, the catchment area surrounding Head Maralla is 450 hectares, with 70 percent of the land used for forest, which is protected by the army and managed by the Forest Department, and the remaining land used for agricultural purposes and heavily influenced by anthropogenic activities. Head Maralla’s irrigation system is made easier by the Irrigation Department. In Head Maralla, two main canals are operational: 1) Maralla Ravi connection (water flow 22000 Cs) and 2) upper Chenab canal (water flow 16850 Cs). The old canal system was built between 1905 and 1912, while the Head Maralla was built between 1965 and 1968, with 66 gates for water management and balancing.

### Ethnographic data of Head Maralla

The region of Head Maralla is divided between two religious communities, with Muslims making up the majority and Christians making up the minority. Herbal remedies are used by people of many ethnic groups to treat a variety of diseasees. All castes/tribes are represented in Head Maralla, including Jutt, Gujjar, Sheikh, Mughal, Nai, Faqir, Rajput, Malik, and Syed. According to the local government, around 5,000 people reside in the Head Maralla area, with 70% relying on agriculture. The average caste/tribe percentage distribution is as follows: Jutt 40%, Gujjar 20%, Syed 10%, Mughal 10%, Malik 10%, Christian 5%, and others 5%.

### Data collection

For collect data, the following procedures were used: a) surveys, b) informant selection and ethnobotanical knowledge discovery, c) photography and inventory, d) preservation and taxonomic verification, e) botanical identification, and f) quantitative ethnobotanical data analysis. Six trips were planned during the summer and winter, focusing on the monsoon season, when the greatest plant diversity was available and local inhabitants were notified. After several field trips and gathering information on respondents and their traditional knowledge competency, sites were chosen. There is a strong culture of collaboration and hospitality among students and faculty members in the region, so meeting individuals and gathering information for research objectives was not a problem after receiving permission from the irrigation and forest departments. Women’s husbands and/or siblings were asked to help them in order to maintain cultural conventions, as most women dislike talking to strangers. Punjabi and Urdu were the languages of communication. The data was collected from all four seasons. Along with local residents, numerous hakims, practitioners, and healers were contacted and discussions regarding various plants, their collecting techniques, and recipes. To gather indigenous knowledge, a rapid appraisal technique (RAA) was used. The survey used Ashebo’s technique of direct engagement with indigenous people through group talks, corner meetings, and semi-structured interviews [34].

For interview, questionnaire was divided into two sections: a) demographic information and b) plant usage. Medicinal and industrial plants were then separated from the various applications. Traditional knowledge was recorded as an inventory, which included local plant names, components utilised, preparation techniques, mode of use, and diseasees treated (questionnaire as S1 File). Photographs of various places, vegetation, and some of the sites’ distinctive flora were taken with cameras "Cannon D 700" and "Sony cyber shot" for identification. After comparing the data to the literature, an inventory was created. Local culture, customs, and flora, and general demographic information were documented.

#### Documentation and identification of plant

From February 2017 to August 2019, ethnobotanical data and plants were gathered. The plants were pressed and treated with 1% HgCl_2_ solution and then mounted on herbarium sheets in the Department of Botany, University of Gujrat, Gujrat, Pakistan. Collected species were recognised and compared to the Flora of Pakistan as well as existing literature, while complex specimens were confirmed with the Quaid-i-Azam University collection in Islamabad, Pakistan [17]. During field surveys, identification was based on native plant names and the assistance of local informants. The Flora of Pakistan (http://www.efloras.org/index.aspx) was used for taxonomic confirmation. APG IV (where appropriate), the USDA plant database, and ‘The Plant List’ were also used to double-check accurate categorization and nomenclature. For proper botanical name confirmation, the majority of the names are based on ‘The Plant List’ (http://www.theplantlist.org).

### Quantitative analyses of ethnobotanical data

#### Informant’s consensus factor

The Informants consensus factor (F_ic_) was computed to evaluate the usage of medicinal plants and their discovery of bioactive chemicals, which is the most commonly used technique [35]. This approach was used to locate and highlight information on specific type of disease groups. The link between the "number of used reports in each category (Nur) minus the number of species utilised (nt)" and the "number of used-reports in each category minus 1" is estimated using this tool. The low score around 0 indicates that the plants were picked at random for a few or a single ailment, or that the informant did not provide information about plant use [36]. F_ic_ wascalculated using the following formula.


$$Fic=\frac{Nur-Nt}{Nur-1}$$

#### Cultural Significance Index (CSI)

Cultural significance index (CSI) is the relationship among use reports of a given species and agreement between the informant’s knowledge. It was calculated by following formula [37].

CSI=∑(i×e×c)×CF

Where *i* is the management of species having significant effect on community (a species cultivated, functioned by any mean is presented score of 2 and the value 1 is presented if species is free from any kind of manipulation), *e* is use for the preference of the informants for one species over another plant species for particular purposes, *c* is use frequency of species. Correction factor (CF) is the level of informants consensus which derives from plant species citation divided by the number of citation of the most mentioned plant species.

#### Relative Frequency of Citation (RFC)

RFC is the priority order between the listed plant species and its value is depended on the numbers of participants who have mentioned a specific plant species as indicating its importance. The RFC was assessed by following formula [38]:

RFC=FC/N(0<RFC<1)

Where, FC is the number of participants which are stated specific species as a good medicinal plant and N is the total number of participants who involved in the study.

#### Use Value (UV)

UV was calculated by applying standard described earlier [39];

UV=U/n

Where U is the total number of use reports cited by informants for a specific plant and n is the total number of informants interviewed for a given plant species.

#### Comparison with neighboring areas

A comprehensive study was carried out to compare current findings to previously published data. Fourty studies were deemed to be the most appropriate for comparing area, research year, families, total species common in both regions, plants with comparable uses (%), plants with contrasting uses (%), species enrolled in defined area, and citation. By assessing the reported species and their medicinal significance, the current study was compared to previously published data in different parts of the world using the Jaccard index [40].


JI=c×100/a+b-c

#### Pearson correlation

Correlation between different parameters such as CSI, RFC and UVs were traced using Pearson’s correlation using R packages (v.3.6.1) by using ggpubr (https://cran.r-project.org/web/packages/ggpubr/index.html) package to confirm the significant differences.

## Results and discussion

### Demography of respondents

A total of one hundred local informants were formally approached for the data, with informants ranging in age from 40–50, 51–60, 61–70, 71–80, and >80 years old. There were 73 men and 27 women among the 100 informants. While 15 were traditional healers (hakims), others had professional ties to agriculture, fishing, housewives, local government, and workers of the forest, irrigation, and agricultural agencies (Table 1). Although people of different age groups had knowledge, but elders proved more authentic with command in traditional knowledge. Interestingly, other people knew such prominent elders and advised to contact them. A constant contact with the local people was maintained throughout the study to ensure the robust validity of traditional knowledge. Similar results were stated in the studies conducted in Bangladesh [45], Pakistan [46] and India [51].

**Table 1:** Demographic data of informants recorded at Head Maralla.

Age group	Informants	Male	Percentage	Female	Percentage
40–50	14	10	13.69	04	14.81
51–60	22	15	20.54	07	29.97
61–70	33	24	32.87	09	33.31
71–80	26	20	27.39	06	27.22
>80	05	04	5.47	01	3.70
Total	100	73		27	
Educational background		levels		Informants	
Illiterate or primary pass (5 years)		School		42	
Middle pass (8 years)		Middle School		07	
Matric (10 years)		High School		21	
Undergraduate (14 years)		College		21	
Graduate (16 years) or above		University		09	

### Plant diversity

At Head Maralla, 119 different plant species from 54 different groups were recorded (Table 2). There are 88 dicot species, 12 monocot species, 11 aqauatic plants, 5 ferms, and 4 bryophytes among them (Fig 3). Herbs were the most common source of medicine in the region (73 species), followed by trees (22 species), weeds (11 species), shrubs (9 species), foliose (2 species), and thaloids (2 species) (Fig 3). Because of the abundance of herbaceous plants in their surroundings, indigenous people frequently utilise herbs [43]. Lakes, ponds, and ditches in the region were also investigated for aquatic flora and medicinal applications. The most common genera discovered in the water bodies were *Nelumbium*, *Typha*, and *Ceratophyllum*. *Typha* has been found to be widely used by the locals for a variety of uses in several areas. *Marchantia polymorpha* L., *Riccia cavernosa* Hoffm., *Polytricum* sp., and Funaria hygrometrica Hedw. were common bryophytes in the region, while *Osmunda regalis* was a common fern. A floral inventory was developed and presented in Table 2. Presence of common genera including *Ipomoea*, *Euphorbia*, *Ficus*, *Solanum*, *Acacia* and *Amaranthus* were recorded at all sites.

**Fig 3:** Summary of floral diversity recorded at Head Maralla.

**Table 2:** Inventory of wild plants with medicinal and industrial uses along with locality reported from Head Maralla.

S. No.	Botanical Name	Family	Vou. No.	RT	UC	RMT	BLP	Local Name	Locality	Habit	Plant part used	Uses
**Dicotyledons**												
1	*Justicia adhatoda* L.	Acanthaceae	UOG 323	**+**	**+**	**-**	**+**	Baker/Arusa	RT	Shrub	Whole plant	It is used for cure lungs diseases.
2	*Trianthema portulacastrum* L.	Aizoaceae	UOG301	**-**	**+**	**+**	**+**	Itsit	UC	Herb	Whole Plant	The whole plant is effective in liver and lungs problems. It is also considerd a good fodder and vegetable.
3	*Trianthema triquetra* Rotter & Willd.	Aizoaceae	UOG302	**-**	**+**	**+**	**+**	Jangli itsit	RMT	Herb	Whole Plant	It is used in chronic fever, ulcer, as wound healer and fodder.
4	*Achyranthes aspera* L.	Amaranthaceae	UOG317	**+**	**+**	**+**	**+**	Puth Kanda/Chaff Plant	BLP	Herb	Whole Plant	The plant is used against kidney stome. Powder mixed with honey is effective for pneumonia.
5	*Alternanthera pungens* Kunth	Amaranthaceae	UOG320	**+**	**+**	**-**	**-**	Waglon	UC	Herb	Leaves and Fruits	It is used in itching.
6	*Amaranthus graecizans* L.	Amaranthaceae	UOG321	**+**	**-**	**-**	**+**	Phulari	RT	Herb	Leaves	Urination and inflammatory conditions are treated with this drug.
7	*Amaranthus viridis* L.	Amaranthaceae	UOG318	**+**	**+**	**-**	**+**	Chuli	UC	Herb	Whole plant	Fever, kidney pain, hepatitis, and jaundice are treated with it. Leaves are used to cure joint pain and as feed for animals.
8	*Atriplex laciniata* L.	Amaranthaceae	UOG316	**+**	**-**	**-**	**-**	Danywali booti	BLP	Herb	Leaves	Leaves are used in nervous disorder.
9	*Chenopodium album* L.	Amaranthaceae	UOG329	**+**	**+**	**+**	**+**	Bathu	RT	Herb	Whole plant	Roots are used for jaundice and worms. Leaves are used as vegetables and feed for animals.
10	*Chenopodium murale* L.	Amaranthaceae	UOG330	**+**	**+**	**-**	**+**	krund	UC	Herb	Whole plant	Whole plant poweder is taken internally for internal worms and to boost sexual power. The plant is good source of food.
11	*Digeria arvensis* Forssk.	Amaranthaceae	UOG319	**-**	**+**	**+**	**+**	Sessile joyweed, tandla	UC	Herb	Leaves	As a pain reliever and diuretic, it is useful for headaches and burns.
12	*Scandix pectin- veneris* L.	Apiaceae	UOG324	**-**	**-**	**+**	**-**	Marli ajwan	RT	Herb	Flower and leaf	It is used as cooked and in flavoring.
13	*Calotropis procera* (Aiton) Dryand.	Apocynaceae	UOG322	**+**	**+**	**+**	**+**	Akk	UC	Shrub	Whole Plant	Expectorant, purgative, and anthelmintic are all properties of this plant. Latex is used in the treatment of skin diseases and dropsy. The leaves are used to treat discomfort and swelling in the joints, while the powder is used to treat diarrhoea and lungs diseases.
14	*Cleome viscose* L.	Brassicaceae	UOG 326	**+**	**-**	**+**	**-**	Sticky spider flower	RMT	Herb	Seeds, root and	The seeds are anthelmintic and carminative.
15	*Lepidium didymus* L.	Brassicaceae	UOG325	**+**	**+**	**+**	**+**	Lesser swine- cress	BLP	Herb	Whole Plant	The plant is anti-inflammatory, wound healer and fodder.
16	*Cannabis sativa* L.	Cannabaceae	UOG336	**+**	**+**	**+**	**+**	Bhang, Indian Hemp	BLP	Shrub	Whole plant	The plant is used for stomachae and narcotic.
17	*Cichorium intybus* L.	Compositae	UOG 315	**+**	**-**	**-**	**-**	Kashni	BLP	Herb	Whole Plant	The plant is effective in constipation and headache.
18	*Carthamus oxyacantha* M. Bieb.	Compositae	UOG310	**+**	**+**	**+**	**+**	Poli/Carth amus	BLP	Herb	Seeds	Oil extracted from seed is effective against ulcer, toothaches, and skin.
19	*Artemisia scoparia* Waldst. & Kitam.	Compositae	UOG305	**+**	**+**	**+**	**+**	Jahu	RMT	Herb	Whole Plant	The plant has aesthetic value and is used for skin ailments.
20	*Eclipta prostrata* (L.) L.	Compositae	UOG307	**+**	**+**	**+**	**-**	Sofed Banghra	BLP	Herb	leaves	Allergies, athlete’s foot, and ringworm are all treated with leaf paste. It’s also used to treat urticaria and blood purification.
21	*Erigeron bonariensis* L.	Compositae	UOG314	**+**	**+**	**-**	**-**	Horse weed	RMT	Herb	Whole plant	Diarrhoea, bleeding, and haemorrhoids are all treated with this medicine. Dysentery and diabetes are treated using the leaves.
22	*Erigeron canadensis* L	Compositae	UOG313	**+**	**-**	**+**	**+**	Horse weed	UC	Herb	Whole Plant	Internal bleeding and bleeding piles are treated with this medication. Diarrhea, diabetes, and dysentery are all treated using leaves.
23	*Parthenium hysterophorus* L.	Compositae	UOG311	**+**	**+**	**+**	**+**	White top weed	RT	Shrub	Seed, leaves and bark.	It’s used to treat skin problems and is frequently used internally as a treatment for a variety of ailments‥
24	*Silybum marianum* (L.) Gaertn.	Compositae	UOG312	**-**	**+**	**-**	**+**	Milk thistle	BLP	Shrub	Fruit and leaves	The plant is used jaundice, chronic irritation, and in heart burn.
25	*Sonchus asper* (L.) Hill	Compositae	UOG309	**+**	**-**	**+**	**+**	Spiny sow Thistle	RT	Herb	Whole plant	Plant powder is used for healing of wound.
26	*Xanthium strumarium* L.	Compositae	UOG306	**+**	**+**	**+**	**+**	Chota Dha tura/Cocklebur	UC	Shrub	Roots and fruit	It’s used to treat gastrointestinal problems, as a demulcent, for smallpox, and as an antimalarial. It’s also used to treat TB and renal problems.
27	*Tinantia erecta* (Jacq.) Fenzl	Commelinaceae	UOG331	**+**	**-**	**-**	**-**	Peli booti	BLP	Herb	Flowers and Leaves	It’s used to cure coughs, nosebleeds, and diarrhoea, as well as cancer cells‥
28	*Convolvulus arvensis* L.	Convolvulaceae	UOG334	**+**	**+**	**+**	**+**	Lehli	RT	Herb	Whole Plant	Constipation, headaches, wound healing, and menstruation bleeding are all treated with this plant.
29	*Cuscuta reflexa* Roxb.	Convolvulaceae	UOG 338	**-**	**-**	**+**	**-**	Akash bail/Dodder	RMT	Herb	Stem	It is used to lower cholesterol levels, treat diabetes, and purify the blood.
30	*Ipomoea carnea* Jacq.	Convolvulaceae	UOG335	**+**	**+**	**+**	**+**	Bush morning glory	UC	Shrub	Whole Plant	Anticancer and anti-oxytoxic qualities, as well as anti-asthma, anti-bug bites, and anti-burn capabilities‥
31	*Ipomoea eriocarpa* R. Br.	Convolvulaceae	UOG332	**-**	**-**	**+**	**+**	Lagacoco zinho	RMT	Herb	Leaves and Roots	Oral extract of the plant is used to treat ulcers, fevers, and cattle wounds in addition to relieving menstruation discomfort.
32	*Ipomoea pes- tigridis* L.	Convolvulaceae	UOG333	**-**	**+**	**-**	**+**	Tiger foot morning glory	UC	Herb	Leaves	The leaves are used to poultice wounds, and the juice is used to cure rabies‥
33	*Cucumis melo* L.	Cucurbitaceae	UOG 339	**+**	**+**	**-**	**-**	Chiber	UC	Herb	Whole Plant	Whole herb is tonic and useful source of food for animals.
34	*Chrozophora tinctoria* (L.) A. Juss.	Euphorbiaceae	UOG 343	**-**	**+**	**+**	**+**	Dhadal	RMT	Herb	Flowers and leaves	It is used for wound healing.
35	*Euphorbia helioscopia* L.	Euphorbiaceae	UOG340	**+**	**+**	**+**	**+**	Gandi buti	UC	Herb	Whole Plant	Latex is applied to eruption. Seeds with pepper are given in cholera.
36	*Euphorbia hirta* L.	Euphorbiaceae	UOG341	**+**	**+**	**+**	**+**	Dudhi	RMT	Herb	Whole Plant	Expectorant, used in bronchial affection, and asthma.
37	*Euphorbia milii* var. splendens (Bojer ex Hook.) Ursch & Leandri	Euphorbiaceae	UOG344	**-**	**-**	**+**	**-**	Dohdak	UC	Herb	whole plant	It’s used as an expectorant to treat coughs and other throat problems.
												Changed Words
												Structural Changes
												Thesaurus

38	*Euphorbia prostrate* Aiton	Euphorbiaceae	UOG342	**-**	**-**	**+**	**-**	Prostrate sandmat	UC	Herb	Whole Plant	Whole herb is used for allergies and internal worms.
39	*Ricinus communis* L.	Euphorbiaceae	UOG345	**+**	**+**	**+**	**+**	Arind/ coaster oil	BLP	Shrub	Leaves and Seeds	Leaves are pain killer and seed help in reducing snake poisonus‥
40	*Leucas aspera* (Willd.) Link	Lamiaceae	UOG354	**+**	**-**	**+**	**+**	Jumka boti	RT	Herb	Whole Plant	Whole herb is used to treat lung and liver problems.
41	*Mentha spicata* L.	Lamiaceae	UOG352	**+**	**+**	**+**	**+**	Podina	BLP	Herb	Whole Plants	Leaves are effective used as a tonic, flatus-relieving, anti-seditious, and digestive.
42	*Mentha longifolia* (L.) L.	Lamiaceae	UOG353	**+**	**-**	**+**	**+**	Jangli podina	UC	Herb	Whole plant	Whole plant is used againt stomachic diseases and as fodder.
43	*Lathyrus aphaca* L.	Leguminosae	UOG348	**+**	**-**	**+**	**-**	Jangli matar	RMT	Herb	Whole plant	The whole herb is used oil extraction and fodder.
44	*Medicago laciniata* (L.) Mill	Leguminosae	UOG349	**+**	**-**	**-**	**+**	Mena	BLP	Herb	Whole plant	Herb is effective in constipation, kidney disorder, and feed for animals.
45	*Melilotus indicus* (L.) All.	Leguminosae	UOG389	**+**	**-**	**+**	**+**	Sinjiee	UC	Herb	Whole plant	Plant is used as bandage on effected parts of skin and for eyes tonic.
46	*Acacia modesta* Wall.	Leguminosae	UOG 355	**+**	**-**	**+**	**+**	Phulai	BLP	Tree	Gum	Gum is a restorative as well as an adhesive that is utilised in a variety of culinary sectors. Also used as grazing animal feed.
47	*Acacia nilotica* (L.) Delile	Leguminosae	UOG356	**+**	**+**	**+**	**+**	Keekar	BLP	Tree	Bark, pods and gum.	Plant extract has astringing properties, barks is effective against diarrhea.
48	*Albizia lebbeck* (L.) Benth.	Leguminosae	UOG357	**-**	**+**	**+**	**+**	Kala sirin	RT	Tree	Bark	Bark is used to treat infertility, hernia and other body parts.
49	*Alhagi maurorum* Medik	Leguminosae	UOG346	**-**	**+**	**-**	**-**	Jawan Janasa booti	RT	Herb	Whole plant	Whole herb is effective in cough, fever, constipation and skin allerigies. Herb is also used as fodder.
50	*Cassia fistula* L.	Leguminosae	UOG327	**-**	**+**	**-**	**-**	Amaltas/ Golden shower	RT	Tree	Whole Plant	Whole plant is used for abdominal pain cough, headache and has blood purifying properties.
51	*Dalbergia sissoo* DC.	Leguminosae	UOG388	**+**	**+**	**+**	**-**	Tali	RMT	Tree	Leaves, root and bark	Stimulant, astringent and alterative.
52	*Senna occidentalis* (L.) Link	Leguminosae	UOG328	**+**	**+**	**+**	**+**	Desi Sanna	RMT	Herb	Whole plant use	Effective against body swelling, leaves are used for piles, lungs and liver treatment.
53	*Tephrosia lupinifolia* DC.	Leguminosae	UOG347	**-**	**-**	**+**	**-**	Fish poison	UC	Herb	Leaves and root.	Leaves and roots are diuretic, aloso used as cure against snake biting and liver diseases.
54	*Trifolium resupinatum* L.	Leguminosae	UOG350	**-**	**+**	**-**	**-**	Jangli shtala	UC	Herb	Whole plant	Whole herb is good source of vegetable and fodder to enhance the production of milk in animals.
55	*Bombax Ceiba* L.	Malvaceae	UOG361	**+**	**-**	**+**	**-**	Sumbal	UC	Tree	Whole plant	Treatment of genital organs, gonorrhea, mordant for looseness
56	*Malva parviflora* L.	Malvaceae	UOG360	**+**	**+**	**+**	**+**	Sonchal	BLP	Herb	Herb Leaves and seed	Herb is used for body shevering, lungs and digestive diseases.
57	*Malva sylvestris* L.	Malvaceae	UOG359	**+**	**+**	**+**	**+**	Khabzi	UC	Herb	Whole plant	Herb has cooling effect, help in reducing fever and is alo used for urinary related problems.
58	*Melia azedarach* L.	Meliaceae	UOG358	**-**	**+**	**-**	**-**	Dherak	RMT	Tree	Leaves and fruit	Leaves and fruits are used for skin allergies.
59	*Morus alba* L.	Moraceae	UOG366	**+**	**+**	**+**	**-**	Sheehtoot	UC	Tree	Fruit and bark	It has cooling effects, effect in throat soring and baki is helpful in removal of body wastes.
60	*Morus nigra* L.	Moraceae	UOG367	**-**	**-**	**+**	**+**	Kala toot	BLP	Tree	Root, leaves and fruit	It is used for stomach diseases.
61	*Broussonetia papyrifera* (L.) L Her. ex Vent.	Moraceae	UOG362	**+**	**+**	**+**	**+**	Jangli toot	UC	Tree	Bark and fruit	The plant help in reducing fever and loosing of facets.
62	*Ficus benghalensis* L.	Moraceae	UOG363	**-**	**-**	**+**	**-**	Borh	UC	Tree	Whole Plant	It is effective against jaundice and increase sex power.
63	*Ficus elastic* Roxb. ex Hornem.	Moraceae	UOG365	**-**	**-**	**+**	**-**	Rubber	RT	Tree	Whole Plant	Leaves are used in liver diseases.
64	*Ficus religiosa* L.	Moraceae	UOG364	**-**	**+**	**-**	**-**	Peepal	BLP	Tree	Fruit and Seeds	It is used to cure lungs, loosening and bladder diseases.
65	*Callistemon viminalis* (Sol.ex Gaertn.) G. Don	Myrtaceae	UOG371	**+**	**+**	**+**	**+**	Bottle brush	BLP	Tree	Whole Plant	The plant is rich source of antioxidants and other chemicals.
66	*Eucalyptus camaldulensis* Dehnh.	Myrtaceae	UOG369	**+**	**+**	**+**	**+**	Sufeda	BLP	Tree	Leaves	Leaves are effective in curing ear, nose and throat infections.
67	*Eucalyptus globulus* Labill.	Myrtaceae	UOG308	+	+	-	-	Chatta Sufeda	UP	Tree	Whole Plant	The plant is used for viral, allerigic and ulcer related problems. Also it is a good source of wood for domistic needs and fragrance.
68	*Eucalyptus tereticornis* SM.	Myrtaceae	UOG368	**+**	**-**	**+**	**+**	Sufeda	RMT	Tree	Leaves	Common cold and nose infections.
69	*Psidium guajava* L.	Myrtaceae	UOG370	**+**	**-**	**-**	**-**	Amrood	RT	Tree	Whole plant	Fruits helps in digestion. Wood is uded for domestic use.
70	*Oxalis corniculata* L.	Oxalidaceae	UOG372	**+**	**+**	**+**	**+**	Khuti booti/Yell	RT	Herb	Whole plant	Antiscorbic, refrigerant, cooling and stomachic.
71	*Anagallis arvensis* L.	Primulaceae	UOG387	**+**	**-**	**+**	**+**	Dahber booti	UC	Herb	Whole plant	The herb is used for reducing fever, loosening and cought.
72	*Fumaria indica* (Hausskn.)	Papaveraceae	UOG351	**+**	**+**	**+**	**+**	Papra	UC	Herb	Whole Plant	It’s used to treat discomfort, a runny nose, and diarrhoea. Dyspepsia, liver illness, and constipation are also treated with this plant.
73	*Polygonum avicularia* L.	Polygonaceae	UOG384	**-**	**+**	**+**	**-**	Spike weed	RT	Herb	Whole Plant	The whole herb is used to reduce cold, headache and also as vegetale.
74	*Polygonum plebeium* R. Br.	Polygonaceae	UOG383	**-**	**+**	**+**	**+**	Cherri hatha, small knotweed	BLP	Herb	Whole Plant	The herb is used in cough, cold stroke and feed for animals.
75	*Rumex crispus* L.	Polygonaceae	UOG386	**+**	**+**	**+**	**-**	Kali palak	BLP	Herb	Whole Plant	It is used to cure digestive diseases and also used as saag and feed for animals.
76	*Rumex dentatus* L.	Polygonaceae	UOG385	**+**	**+**	**+**	**+**	Jangli palak	UC	Herb	Whole Plant.	The herb helps in blod pressure, loosning, and fodder for animals.
77	*Portulaca oleracea* L.	Portulacaceae	UOG373	**+**	**-**	**+**	**+**	Lonak, Kulfa, Purslane	RT	Herb	Whole plant	The whole herb is help in allergic diseases, urinary problems and iron deficiency.
78	*Portulaca quadrifida* L.	Portulacaceae	UOG374	**+**	**-**	**+**	**-**	Desi Kulfa	UC	Herb	Whole plant	The herb is effective to treat lungs related diseases and also used as vegetables.
79	*Ranunculus muricatus* L.	Ranunculaceae	UOG391	**-**	**-**	**+**	**+**	Buttercup	RMT	Herb	Whole Plant	The plant has aesthetic and fodder values.
80	*Ziziphus jujuba* Mill.	Rhamnaceae	UOG390	**+**	**+**	**+**	**-**	Ber		Tree	Leaves and fruits.	The leaves are used on external dog bite and has bitter propterties.
81	*Datura innoxia* Mill.	Solanaceae	UOG394	**+**	**-**	**+**	**+**	Datura/ Thorn Apple	RT	Herb	Seeds	The herb is effective againt It is used in the treatment of stomach diseases and allergies. Also used as poultices, gonorrhea and as a fodder.
82	*Solanum nigrum* L.	Solanaceae	UOG395	**+**	**+**	**+**	**-**	Kainch Mainch Nightshade	BLP	Herb	Leaves	Whole herb is used for body pain and mensturation. Leaves are considered good blood purifier. Leaf extract is used to cure earache.
83	*Solanum xanthocarpum* Schrad. & H. Wendl.,	Solanaceae	UOG392	**-**	**+**	**+**	**-**	Kandiari	UC	Herb	Whole Plant	It is used as antipyretic, abdominal pain and also as fodder.
84	*Withania somnifera* (L.) Dunal	Solanaceae	UOG393	**+**	**+**	**+**	**+**	Ak San/ Winter Cherry	UC	Herb	Whole plant	The whole herb is used for increased sexual ability, fuits are effective for controlling blood pressure, Tuber is used for stomach infection. Plant is also cure high cholesterol.
85	*Tamarix aphylla* (L.) H. Karst.	Tamaricaceae	UOG396	**-**	**+**	**+**	**-**	Frash, Okan, Peelish	RMT	Tree	Whole plant	It is used as stimulant and bitter. It also cures allergic disorders. Timber is used for domestic needs.
86	*Lantana camara* L.	Verbenaceae	UOG398	**+**	**+**	**+**	**+**	Butterfly weed	BLP	Shrub	Stalk & leaves	The extract from leaves is used to cure ulcer. They are also antipyretic and carminative.
87	*Tribulus terrestris* L.	Zygophyllaceae	UOG399	**+**	**+**	**+**	**+**	Bhakra	BLP	Herb	Whole Plant	Whole plant is sex tonic, help in ejaculation, joint disorder and gonorrhea and urinogenital diseases.
**Monocotyledons**												
88	*Phoenix dactylifera* L.	Arecaceae	UOG 303	**-**	**+**	**-**	**-**	Phall wali khajoor	RT	Tree	Leaves, fruit, and stem	The seed is eaten for loosening, tooth pain and fuel.
89	*Phoenix sylvestris* (L.) Roxb.	Arecaceae	UOG 304	**+**	**+**	**-**	**-**	Khajoor	BLP	Tree	Leaves, fruit, and stem	The plant is used for constipation, toothache and domestic purposes.
90	*Cyperus rotundus* L.	Cyperaceae	UOG 337	**-**	**+**	**-**	**-**	Deela	RMT	Herb	Rhizom es	The rhizome is used in reducing fever, lose motions, food infection, and stomach disorder.
91	*Avena sativa* L.	Poaceae	UOG 377	**+**	**-**	**-**	**-**	Javi	UC	Herb	Whole Plant	The herb is used to reduce blood pressure, digestion, fodder and fuel.
92	*Cynodon dactylon* (L.) Pers.	Poaceae	UOG 382	**+**	**+**	**+**	**+**	Khabal	RT	Herb	Whole plant	The whole plant is used in constipation, astringent, and diuretic.
93	*Desmostachya bipinnata* (L.)	Poaceae	UOG 378	**+**	**+**	**+**	**-**	Dabb	RT	Herb	Whole Plant	Whole herb is effective in blood infections and used in domestic purposes.
94	*Dichanthium annulatum* (Forssk.) Stapf	Poaceae	UOG 376	**-**	**-**	**-**	**+**	Palwangrass	blp	Herb	Whole Plant	The whole plant is utilized for domestic side.
95	*Eleusine indica* (L.) Gaertn.	Poaceae	UOG 380	**-**	**-**	**+**	**-**	Crow feet grass	RT	Herb	Whole Plant	The plant is used in constipation, blood, digestive problems.
96	*Poa annua* L.	Poaceae	UOG 379	**-**	**-**	**+**	**-**	Chota grass	RMT	Herb	Whole Plant	The herb effective in constipation, and burning sensation.
97	*Saccharum arundinaceum* Retz.	Poaceae	UOG 381	**+**	**+**	**+**	**-**	Sarkanda	BLP	Herb	Stem and root	The herb is used for controlling blood pressure and excess release of urine.
98	*Saccharum spontaneum* L.	Poaceae	UOG 375	**+**	**+**	**+**	**+**	Kahi	RT	Herb	Whole plant	The whole plant is use against TB and blood disease.
99	*Typha latifolia* L.	Typhaceae	UOG 397	**+**	**+**	**+**	**-**	Large marsh	RMT	Herb	Leaves and Pollens	Astringent, sedative and anticoagulant.
**Ferns**												
100	*Equisetum arvense* L.	Equisetaceae	UOG 400	**-**	**-**	**+**	**-**	Char booti	UC	Herb	Stem	It is used for the treatment of diabetes.
101	*Marsilea quadrifolia* L.	Marsileaceae	UOG 403	**+**	**+**	**+**	**+**	Four leaf clove	RMT	Herb	Seeds and leaves	The juice extracted from the leaves is used in reducing blood pressure, reduce swellings, fever and snake biting.
102	*Osmunda regalis* L.	Osmundaceae	UOG 401	**+**	**+**	**+**	**-**	Spiral booti	BLP	Herb	Roots and shoots	The roots and leaves are blood and kidney disorders
103	*Adiantum capillus-veneris* L.	Pteridaceae	UOG 402	**-**	**-**	**+**	**-**	Maiden hair fern	RT	Herb	leaves	The wole herb is used in lung diseases.
104	*Azolla pinnata* R. Br.	Salviniaceae	UOG 418	**+**	**-**	**+**	**+**	Mosquito fern	RMT	Herb	Whole plant	Whole herb is considered as a good pollution removal from environment.
**Bryophytes**												
105	*Funaria hygrometrica* Hedw.	Funariaceae	UOG 416	**+**	**+**	**+**	**+**	Moss	UC	Foliose	Whole Plant	Plant is used to cure heart and brain diseases.
106	*Marchantia polymorpha* L.	Marchantiace ae	UOG 415	**+**	**-**	**+**	**-**	Umbrella liverwort	BLP	Thalloid	Whole Plant	The plant is used to control blood pressure and jaundice.
107	*Polytricum* sp.	Polytrichaceae	UOG 417	**+**	**-**	**+**	**+**	Hair moss	RT	Foliose	Whole Plant	The plant is effective againt lung diseases.
108	*Riccia cavernosa* Hoffm.	Ricciaceae	UOG 418	**+**	**-**	**+**	**+**	Sponswat ervorkje	BLP	Thalloid	Whole Plant	Whole plant is effective again urination and eyes problems.
**Aquatic Plants**												
109	*Pistia stratiotes* L.	Araceae	UOG 405	**+**	**-**	**+**	**-**	Water lettuce	RT	Weed	Leaves	Leaves are rich in antioxidant.
110	*Spirodela polyrhiza* (L.)	Araceae	UOG 404	**+**	**+**	**-**	**-**	Duckweed	RT	Weed	Whole Plant	Whole plant is used for wound healing.
111	*Ceratophyllum demersum* L.	Cerotaphyllaceae	UOG 406	**+**	**-**	**+**	**-**	Coontail Weed	RT	Weed	Leaves	Leaves are effective in bile secretion and scorpion bites.
112	*Chara Schweinitzii* A. Braun	Charophyceae	UOG 407	**+**	**+**	**-**	**+**	Musk grass	BLP	Weed	Stem, Branche s	The leaves are antiseptic.
113	*Hydrilla verticillata* (L.F.) Royle	Hydrocharita ceae	UOG 414	**-**	**+**	**+**	**+**	Esthwaite waterweed	RMT	Weed	Leaves	The paste made from leaves has healing properties and in the abscess boil.
114	*Nelumbium nuciferum* Gaertn	Nymphaeaceae	UOG 409	**+**	**+**	**+**	**-**	Indian lotus	UC	Weed	Whole Plant	The plant is used for heart and liver disorder and piles.
115	*Nymphaea lotus* L.	Nymphaeaceae	UOG 408	**+**	**+**	**-**	**-**	Water lily	RT	Weed	Leaves	Leaves help in menses and stomach disorder.
116	*Eichhornia crassipes* (Mart.)	Pontederiaceae	UOG 410	**+**	**+**	**+**	**+**	Water hyacinth	BLP	Weed	Petiole and leaves	It is antioxidant, carotene rich and used as manure.
117	*Potamogeton* sp.	Potamogeton aceae	UOG 412	**+**	**-**	**-**	**-**	Pond weed	UC	Weed	Leaves and seeds	Leave and seeds are used in stomach diseases and flavoring.
118	*Zannichellia palustris* L.	Potamogetonaceae	UOG 411	**+**	**-**	**+**	**-**	Horned pondweed	RT	Weed	Leaves	Leaves are effective in digestion and other digestive diseases.
119	*Spirogyra buchetii* Petit	Zygnemataceae	UOG 413	**-**	**+**	**+**	**+**	Green algae	BLP	Weed	whole Plant	The plant is rich in antioxidant and mutagenic.

Vou. No. Voucher Number; RT, River Tavi; UC, Upstream Chenab; RMT, River Munawarwala Tavi; BLP, Bhalolpur. Signs used are as indication of presence (+) or absence (-) of particular species at particular location.

### Plant part (s) used in major disease categories

The availability of plant parts and local knowledge have a role in the usage of plant parts in the production of recipes. As shown in Fig 4, the whole plant was the most commonly used part of the plant, accounting for 55 percent of applications in both traditional herbal medicine and industrial applications, followed by leaves (28%), seeds (6.7%), fruits (5.9%), bark (5%), roots (4.2%), stems (3.3%), flowers (2.5%), and gums (2.5%) (1.6%). Fig 5 shows that urine (14% spp.), cough (8.4% spp.), cold (6.7% spp.), asthma and stomach diseasees (5.95% spp.), constipation, and skin infections (5%spp.), and diarrhoea (5% spp.) were all utilised as fodder (4.2% spp.). The local inhibitants like to utilise the entire plant because most of the flora was herbaceous in nature [41, 42]. Apart from the entire plant, the leaves are the most important photosynthetic organ. Similarly, leaves are simple to collect and are rich in health beneficial secondary metabolites which contribute significantly to the treatment and prevention of health disorders [33, 43, 44]. Previous research has shown leaves as one of the most often utilised plant parts for grazing and therapeutic uses [45, 46].

**Fig 4:** The percentage of different parts of plants used for ethnomedicine.

**Fig 5:** Multipurpose uses of native plants for domestic and medicinal utilities.

### Local community health and wellbeing

Wild plants have been reported to have the ability to treat a variety of life-threatening diseasees, including ulcers, tumours, diarrhoea, and asthma. Similarly, the usage of wild plants for medicinal and aromatic reasons has been reported in many parts of the nation; nevertheless, there is a pressing need to investigate the potential on a scientific basis. Concentrated efforts would be necessary in this respect, and community mobilisation for the conservation of local wild plant resources is proposed [47]. Studies conducted in Mardan KPK reported species such as *Morus alba* L., *Luffa cylindrical* L. (Rox), and *Fagonia cretica* L., for medicinal and food purposes [48].

Antimicrobial properties have been linked to several species, as well as therapeutic benefits against a variety of ailments. These plants have also been reported in Pakistan (Khyber Pakhtun Khwa, Punjab North, and Azad Jammu and Kashmir) [48]. Screening for possible antimicrobial agents is obviously necessary before assessing therapeutic potential and isolating novel bioactive compounds [49]. A research based on ethnobotanical data from Morgah Biodiversity Park in Rawalpindi, Pakistan, found that local residents benefit from 40 species belonging to 39 genera and 32 families [50].

Furthermore, changes in lifestyle have altered living as a result of the availability of alternatives to indigenous plants, which has resulted in a decline in herbal use. As a replacement for natural goods, a variety of synthetic materials are available on the market. Similarly, furniture constructed of wood, especially from *Delbergia sessio* DC., has been replaced by synthetic materials such as plastic, iron, plywood, and so on. The low demand for such furniture and houses is attributable not just to a scarcity of raw materials, but also to their expensive cost. Surprisingly, Gujrat and Chiniot areas are still known in Pakistan for furniture manufacture and lure European markets. Windows and doors made of *Cedrus deodara* (Roxb.) D. Don., are also very popular but cost raises many folds. As a result, the younger generation is gravitating toward synthetic materials. Furthermore, Sialkot is well-known for producing sporting goods and musical instruments, but it has recently turned its focus to alternative materials. Cutting down trees and reducing forest timber and lumber capacity are two strong reasons for the lack of ability to support local industry. Such paradigm shift complies with documenting ethnobotanical knowledge of the concerned area. It is therefore important to document the ethnobotanical data before the information is lost.

### Quantitative analysis of ethnobotanical data

#### Informant consensus factor (F_ic_)

The F_ic_ was estimated for 11 different diseases, including respiratory diseases, throat illness, liver disease, digestive system, constipation, wound healing, renal disorders, jaundice, fever, diarrhoea, inflammatory issues, and constipation. The F_ic_ for these 11 illnesses varied from 0.73 to 0.93, with 0.73 indicating inflammatory issues and 0.93 indicating respiratory issues. The average F_ic_ was 0.87, indicating that the informants were in agreement on the usage of plants to cure a certain disease. The order of F_ic_ (Table 3) was documented for respiratory disorders (0.93), throat disease (0.92), liver disorders (0.86), digestive system (0.84), constipation (0.75), wound healing (0.83), kidney disorder (0.81), jaundice (0.79), fever (0.75), diarrhea (0.74), and inflammatory problems (0.73). Respiratory disorders were most persistent in the study area. The local people were using 10 different species. The low F_ic_ value was recorded for inflammatory problems (0.73), diarrhea (0.74) and fever (0.79). Low values might be attributed to a lack of communication between informants. The highest value, near to 1, showed that people were utilising these species in significant amounts, whilst the lowest value indicated that informants disagreed on the utility of these species in the treatment of various diseases.

**Table 3:** Disease category cured through number of taxa/species, reports and informants consensus factor (ICF) for Head Maralla vegetation.

Use categories	Number of taxa/species Nt/s	Number of use reports Nur	ICF
Respiratory disorders	3	32	0.93
Throat diseases	3	29	0.92
Liver disorders	5	31	0.86
Digestive system	7	34	0.84
Constipation	14	53	0.75
Wound healing	6	31	0.83
Kidney disorders	6	28	0.81
Jaundice	7	30	0.79
Fever	8	30	0.75
Diarrhea	8	28	0.74
Inflammatory problems	9	31	0.73

The effectiveness of F_ic_ for disease treatment is mostly determined by the availability of plant species in the region [35]. These species have also been reported from other parts of Pakistan [36–40]. *Adiantum capillus-veneris* L.; leaf decoction is effective for lung diseases in the Murree region and *Cichorium intybus* L., root and leaves used against blood pressure and digestive diseases in the district Bagh, Azad Kashmir [40, 41].

Respiratory and throat ailments were frequent in the study area, which might be connected to a shortage of hygienic food and drinking water [51, 52]. Because active chemicals may be found in plants, they are frequently used to treat such illnesses. Several ethnic cultures throughout the world employ traditional knowledge to treat respiratory and throat disorders [23, 35, 36]. According to ethnopharmacological inquire about, respiratory infections and throat sicknesses are categorised as ß in numerous parts of the world [32, 53]. In spite of the fact that Head Maralla has never been considered ethnobotanically or ethnomedically, the current discoveries are reliable with past reports from adjacent regions [36, 54], especially supporting the findings of Kayani et al, 2014 [16], who found that respiratory disarranges and throat contaminations were the foremost common maladies in Gallies of Abbottabad, a city within the Himalayan run of Northern Pakistan.

In this study, high F_ic_ values suggested that informants were very reliant on medicinal plant usage, particularly for symptoms of respiratory illnesses and throat diseasees, but low F_ic_ values for constipation indicated that informants had little understanding [55]. A high ICF value is often associated with a small number of specific plants with high use reports for treating a single disease category, whereas low values are associated with a large number of plant species with nearly equal or high use reports, implying a low level of agreement among informants or the use of reported plant species to treat a specific disease category [56].

#### Cultural Significance Index (CSI)

The cultural importance index is used to determine the value of a particular plant that is used by the locals. In CSI, species identification is linked to their usefulness for humans and is seen as a secondary component in the cultural recognition of a plant [42]. The cultural importance of a species has been shown to differ among local populations. For example, CSI values range from 0.12 to 7.55, and are heavily influenced by locals’ preferences and frequency of usage (Table 4). This is probably influenced by the level of information, the cultural backgrounds, and the prevailing conditions in the areas. The highest CSI value was found for *Adhatoda*. *vesica* (7.55) which is extensively used in respiratory disorders and in digestive problems. Some other species such as *A*. *nilotica* (6.71), *Acacia modesta* (6.13) were highly cited by informants to be used in various applications. Plants’ cultural relevance is measured by their frequency, quality preferences, and therapeutic applications. The high CSI values of plant species also demonstrate that the more a species is available to community members for therapeutic purposes, the more valuable it becomes. *A*. *vesica*, for example, is a well-known plant that is listed in the Ayurvedic herbal system. It has been used to treat a variety of respiratory, intestinal, and bacterial infections [43]. Furthermore, species defined as having significant cultural importance are not limited to a single location or region, but also extend to other ethnic groups throughout the world. As a result, linked information has been passed down down the generations through experience. *E*. *Canadensis* (0.12), *E*. *bonariensis* (0.15), and *E*. *milii* (0.18) were less popular in the society and hence have a low CSI value. The findings of our investigation are consistent with those of Wong [41].

**Table 4:** Plants with frequency of citations (FC), relative frequency of citations (RFC), use value (UV) and cultural significance index (CSI) values.

Plants Species	FC (n)	RFC	UV	CSI	Plant Species	FC(n)	RFC	UV	CSI
*Acacia modesta* Wall.	50	0.67	0.54	6.13	*Ipomoea carnea* Jacq.	53	0.18	0.87	1.05
*Acacia nilotica* Delile	110	0.25	0.20	6.71	*Ipomoea eriocarpa* R. Br.	79	0.67	0.39	0.28
*Achyranthes aspera* L.	60	0.33	0.47	0.56	*Lantana camara* L.	34	0.37	0.25	3.13
*Adhatoda vesica* L.	65	0.89	0.30	7.55	*Lathyrus aphaca* L.	39	0.73	0.30	2.87
*Adiantum capillus- veneris* L.	90	0.64	0.12	1.34	*Leucas aspera* (Willd.) Link	40	0.74	0.34	0.78
*Albizia lebbeck* (L.) Benth	95	0.32	0.88	2.81	*Medicago laciniata* (L.)	41	0.31	0.31	1.66
*Alhagi maurorum* Medik	50	0.63	0.74	0.36	*Malva parviflora* L.	40	0.46	0.26	0.88
*Alternanthera pungens* Kunth	70	0.20	0.65	2.72	*Malva sylvestris* L.	58	0.85	0.40	0.34
*Amaranthus graecizans* L.	40	0.71	0.76	0.90	*Marchantia polymorpha* L.	44	0.54	0.45	0.49
*Amaranthus viridis* L.	95	0.36	0.16	2.13	*Marsilea quadrifolia* L.	66	0.19	0.35	0.87
*Anagallis arvensis* L.	60	0.34	0.18	1.88	*Melia azedarach* L.	78	0.56	0.25	0.57
*Artemisia scoparia* Waldst. & Kitam.	66	0.63	0.10	0.56	*Melilotus indicus* (L.) All.	56	0.16	0.16	0.75
*Atriplex laciniata* L.	88	0.67	0.15	2.89	*Mentha longifolia* (L.) L.	34	0.26	0.15	0.55
*Avena sativa* L.	90	0.74	0.24	2.77	*Mentha spicata* L.	57	0.54	0.13	1.88
*Bombax ceiba* L.	98	0.45	0.47	1.78	*Morus alba* L.	35	0.18	0.10	0.21
*Broussonetia papyrifera* (L.) L Her. ex Vent.	67	0.43	0.76	3.89	*Morus nigra* L.	67	0.55	0.14	0.60
*Callistemon viminalis* (Sol.ex Gaertn.) G. Don	78	0.55	0.56	1.78	*Nelumbium nuciferum* Gaertn	56	0.45	0.23	0.34
*Calotropis procera* (Aiton) Dryand.	87	0.87	0.56	2.13	*Nymphaea lotus* L.	45	0.71	0.20	0.25
*Carthamus oxyacantha* M. Bieb.	93	0.65	0.56	1.23	*Osmunda rejalis* L.	39	0.17	0.22	2.61
*Cannabis sativa* L.	94	0.65	043	3.67	*Azolla pinnata* R. Br.	35	0.34	0.33	0.19
*Cassia fistula* L.	80	0.80	0.65	0.87	*Oxalis corniculata* L.	58	0.26	0.35	0.56
*Senna occidentalis* (L.) Link	86	0.35	0.61	3.46	*Parthenium hysterophorus* L.	63	0.18	0.36	0.89
*Ceratophyllum demersum* L.	76	0.50	0.26	0.56	*Phoenix dactylifera* L.	45	0.22	0.29	0.78
*Chara Schweinitzii* A. Braun	83	0.54	0.16	0.57	*Pistia stratiotes* L.	78	0.75	0.20	0.18
*Chenopodium album* L.	80	0.83	0.78	2.21	*Poa annua* L.	56	0.57	0.14	4.67
*Chrozophora tinctoria* (L.) A. Juss.	96	0.54	0.75	3.22	*Polygonum plebeium* R. Br.	77	0.63	0.77	0.27
*Cichorium intybus* L.	26	0.38	0.35	1.22	*Polygonum avicularia* L.	67	0.53	0.37	0.18
*Cleome viscose* L.	48	0.19	0.37	0.38	*Polytricum* sp.	56	0.60	0.05	0.17
*Convolvulus arvensis* L.	70	0.58	0.30	0.29	*Portulaca oleracea* L.	45	0.69	0.38	0.78
*Erigeron canadensis* L.	62	0.84	0.21	0.12	*Portulaca quadrifida* L.	38	0.56	0.53	1.19
*Erigeron bonariensis* L.	67	0.19	0.15	0.15	*Potamogeton* sp.	43	0.61	0.20	0.70
*Lepidium didymus* L.	76	0.60	0.11	1.27	*Psidium guajava* L.	30	0.70	0.28	2.33
*Cucumis melo* L.	88	0.70	0.49	3.55	*Ranunculus muricatus* L.	45	0.65	0.34	0.71
*Cuscuta reflexa* Roxb.	56	0.19	0.40	0.38	*Riccia cavernosa* Hoffm.	56	0.70	0.27	0.78
*Cynodon dactylon* (L.) Pers.	59	0.60	0.36	1.44	*Ricinus communis* L.	38	0.92	0.90	1.45
*Cyperus rotundus* L.	88	0.56	0.55	1.16	*Rumex crispus* L.	40	0.20	0.10	1.34
*Dalbergia sissoo* DC	75	0.33	0.28	0.35	*Rumex dentatus* L.	55	0.55	0.17	1.98
*Datura innoxia* Mill.	67	0.40	0.72	0.45	*Saccharum arundinaceum* Retz.	49	0.33	0.45	0.70
*Desmostachya bipinnata* (L.)	88	0.30	0.67	2.11	*Saccharum spontaneum* L.	40	0.84	0.28	1.55
*Chenopodium murale* L.	78	0.15	0.29	0.16	*Ipomoea tigridus*	35	0.26	0.25	0.77
*Dichanthium annulatum* (Forssk.) Stapf	56	0.30	0.64	0.31	*Scandix pectin- veneris* L.	55	0.65	0.09	0.30
*Digeria arvensis* Forssk.	69	0.66	0.23	1.43	*Silybum marianum* (L.) Gaertn.	45	0.83	0.08	0.45
*Ipomoea pestigridis* L.	70	0.37	0.50	0.47	*Solanum nigrum* L.	50	0.20	0.43	0.70
*Eclipta prostrata* L.	58	0.21	0.34	0.23	*Solanum xanthocarpum* Schrad. & H. Wendl.,	55	0.55	0.86	0.90
*Eichhornia crassipes* (Mart.)	67	0.18	0.38	0.18	*Sonchus asper* (L.) Hill	40	0.33	0.26	0.30
*Eleusine indica* (L.) Gaertn.	78	0.27	0.19	0.27	*Spirodela polyrhiza* (L.)	34	0.23	0.11	0.77
*Equisetum arvense* L.	89	0.67	0.57	0.75	*Spirogyra buchetii* Petit	39	0.26	0.59	0.89
*Eucalyptus camaldulensis* Dehnh.	67	0.29	0.38	0.35	*Tamarix aphylla* (L.) H. Karst.	40	0.65	0.33	0.98
*Eucalyptus tereticornis* SM	87	0.26	0.19	0.26	*Tephrosia lupinifolia* DC	56	0.87	0.13	1.43
*Euphorbia helioscopia* L.	58	0.41	0.57	0.44	*Tinantia erecta (Jacq*.*)* Fenzl	68	0.20	0.22	0.76
*Euphorbia hirta* L.	89	0.29	0.38	0.30	*Trianthema portulacastrum* L.	55	0.68	0.29	0.58
*Euphorbia prostrate* Aiton	78	0.54	0.18	0.56	*Trianthema triquetra* Rotter& Willd.	67	0.37	0.34	0.76
*Euphorbia milii var*. *splendens* (Bojer ex Hook.) Ursch & Leandri	49	0.17	0.25	0.18	*Tribulus terrestris* L.	88	0.57	0.87	5.34
*Ficus benghalensis* L.	59	0.49	0.20	0.50	*Trifolium resupinatum* L.	30	0.71	0.58	2.21
*Ficus elastic* Roxb. ex Hornem.	61	0.76	0.16	0.88	*Typha lotifolia* L.	50	0.27	0.62	0.32
*Ficus religiosa* L.	34	0.50	0.21	0.54	*Withania somnifera* (L.) Dunal	86	0.52	0.45	0.78
*Fumaria indica* (Hausskn.)	56	0.80	0.11	1.68	*Zannichellia palustris* L.	35	0.31	0.48	0.37
*Funaria hygrometrica* Hedw.	88	0.23	0.16	2.34	*Ziziphus jujube* Mill.	65	0.37	0.25	0.39
*Hydrilla verticillate* (L.F.) Royle	45	0.40	0.03	0.45	*Phoenix sylvestris* (L.) Roxb.	70	0.35	0.09	0.78
*Eucalyptus globulus* Labill	78	0.27	0.27	0.85	*Xanthium strumarium* L.	85	0.33	0.16	2.34

#### Relative Frequency of Citations (RFC) and Use Value (UV)

The importance of each species among local populations in the region, ethnobotanical and primary health care to keep them robust and productive, was described by the relative frequency of citations. It is determined by dividing the number of informants who claim to have used a plant species by the total number of informants who took part in the survey to share their local knowledge [57]. RFC varies from 0.92 to 0.15 in the current research (Table 4). The greater RFC was obtained for *Racinus communis* (0.95), *Adhatoda*. *vesica* (0.89), *Calotropis procera* (0.87), *Saccharum spontenum* (0.84), *Silybum marianum* (0.83). These findings show that species have been known to indigenous culture for a long time, but that owing to a lack of knowledge, the majority of people in various parts of the Head Maralla area were unaware of the therapeutic potential of local flora. Based on the number of usage, the relative frequency of citation indicates the importance of particular species among local people [45].

Plants with high RFC values are advised to be used in biological, pharmacological, and phytochemical investigations for drug development [46]. Furthermore, owing to overharvesting by the local population, such plants must be protected on a priority basis. RFC are highly dynamic since they vary from area to region and are based on local people’s traditional knowledge. Plant species with lower RFC values are well recognised, although they are not always less important [47]. Their low values may reflect the native people’s lack of awareness, particularly among the younger generations, who are unaware of the benefits of these plant species. Use value (UV) is a significant index to recognize the plant species which are widely used among local communities [48]. In the reported studies, use values ranged from 0.03 to 0.90 and species with high UV were *Racinus communis* (0.90), *Albizia lebbeck* (0.88), *Ipomoea carnea* (0.87), *T*. *terrestris* (0.87) and *Solanum xanthocarpum* (0.86) (Table 4). The higher UVs of species indicated their significance in the traditional medicinal system [49], which can be recognized with the fact that they are the main choice of the traditional healers for treating ailments and local inhabitants are familiar with these plants [50]. Species with low UVs were *H*. *verticillate* (0.03) *and S*. *pectin-veneris* (0.09). The low UV of plants may reflect less dispersal of species in the region and low ethnomedicinal value of the informants [50].

High UV values were found in *Lepidium didymus*, *Nelumbium nuciferum*, *Albizzia lebbek*, and *Cyprus rotundus* in the current study. It has been found that plants with high use reports (UR) have high UVs, but plants with fewer URs, as reported by informants, have lower UVs. It has also been documented that plants that are handled in a consistent manner are more physiologically active [58].

UV attributes are important and alter with the changing of a region and, in particular, on the basis of people’s understanding, thus UV values can differ from one location to the next and even within the same area. Plants with a lower UV value, on the other hand, are not always insignificant, inspite, they might showi that the young people in the region are unaware of how to use these plants. Based on this understanding, it is reasonable to conclude that plant usage and related information are at risk of not being passed down to future generations and that this knowledge may finally vanish [59]. With the passage of time, more exploration of natural compounds and their evaluation from different plant species, it is ascertaining that the role of traditional knowledge is still more prevalent and important. At the same time one system of medication may fail and other is luckily available to fill the gap and provide alternative remedy. Another benefit is that ethnobotanical knowledge is now scientifically assessed, validated, and further scientific techniques are being utilised to obtain legitimate findings and pure compoundsto make new ways of medication more effective. It is not an issue of youth, but of communal and societal health in Pakistan, where per capita income is still much below that of developed nations, and people of all faiths consult herbalists, hakims, physicians, and religious experts for all feasible solutions and enhanced health care [59–62]. This revealed that there were differences in most of the cited species and their quantitative values. In a study carried out by Abbasi et al. [60], whereas Bano et al. [63] found that *Hippophae rhmnoides* had the highest usage value (1.64) followed by *Rosa brunonii* (1.47) [64]. These variances are primarily due to the area’s great variation in vegetative and geo-climatic conditions, therefore more neighbouring regions should be explored and direct engagement with local populations should be prioritised.

#### Correlation between ethnobotanical indices

The relationship between ethnobotanical indices i.e., CSI, RFC and UV were found significant at 0.01 (Fig 6). A positive correlation was present between CSI and RFC (r = 0.29), followed by CSI and UV (r = 0.29) while UV and RFC showed less significant (r = 0.07). The positive correlation reflects cultural significance of each species and relative importance of the use of plants. Positive combinations provide way forward for their future uses ethnobotaical as well ethnomedicinal.

**Fig 6:** The scatter plot representing correlation for a) RFC vs SCI, b) UV vs RFC and c) CSI vs UV of the vegetation studied at Head Maralla.

#### Jaccard Index (JI)

The Jaccard Index is the indication of relationship among present study and earlier reports, across areas situated near Haed Maralla, within Pakistan and countries having somewhat same livelihood culture. This helps in unwinding new uses of species for ethnomedicinal purposes due to difference in cultural and ethnography of the area [65]. Findings in the reported studies open new avenues for further understanding of the ethnobotanical traditional knowledge as well opportunities for new products development [66, 67]. To make a comparison, ethnopharmacological and ethnobotanical data from 46 published studies in adjacent areas were examined, with just a few of them including related/same species. Many new species were found with novel applications. The vegetation of the neighbouring districts, including Central, Southern, and Northern Punjab, Sindh, KPK, Baluchistan, Azad Kashmir, including District Bhimber, Iran, India, and Bangladesh, was compared to that of Head Maralla. Data from some African countries were also compared having similar type of geoclimatic and topographic conditions.

A few species were common in many reports that reflects cross-cultural knowledge or frequent exchange of material beyond boundaries in past. Consequently, this exchange of knowledge afterwards converted into traditional medicinal system and was transferred from generation to generation.The JI values varied from 7.14 to 0.14 in contrast to the current research and previous studies from Pakistan (Table 5). The highest JI (7.14) was found with previous report from Samahani valley, Azad Kashmir, Pakistan [65], Western Uganda 6.93 [66], Karak, KPK with 6.32 [48] which reflects that plant species reported from theses areas possess similar type of uses more frequently as compared to other reports. Moreover, it is an indication of the culture that people from these areas have limited access to modern mode of medication. The lowest JI such as 0.34, 0.35, and 0.45 was recorded from Sudhan Gali and Ganga Chotti Hills, District Bagh, Azad Kashmir [67], Erer valley of Babile Wereda Eastern Ethiopia [68], and Samburu Community Wamba, Kenya [69], respectively, that indicates few reports of uses similar type of plant species (low number of common species) in the same vicinity. This is probably depending upon the composition of species and their ultimate phytochemical composition that supports their use. Our study shares the highest number of common species with findings from Samahani valley Azad Kashmir, Pakistan [65], with 72.5% similar uses and 31.5% dissimilar uses (Table 5). Similarly, 50 species are common between our study and a study from Karak, KPK that reported a total of 160 species [48], with 68.2% species having similar uses and 5 species with dissimilar uses.

**Table 5:** Comparison with adjacent regions national as well international reports published.

S. No.	Area of studies	Study Year	Number of recorded plant species	Families	Total species common in both areas	Plant with similar uses (%)	Plants with dissimilar uses (%)	Species enlisted only in study area	Jaccard Index	Citations
1	Wana, South Waziristan, Pakistan	2013	50	30	12	32	68	102	1.59	Ullah et al., 2013 [98]
2	Samhani valley Azad Kashmir, Pakistan	2009	120	46	55	72.5	27.5	84	7.14	Hussain and Chaudhary, 2009 [65]
3	Coastal areas of Pakistan	2014	54	27	14	34.6	65.4	99	1.78	Qasim et al., 2014 [105]
4	Nara Desert, Sindh, Pakistan	2008	6	1	16	41	59	115	2.31	Qureshi and Bhatti, 2008 [11]
5	Kotli AJK, Pakistan	2014	33	25	2	6	94	116	0.23	Amjad and Arshad, 2014 [106]
6	Khunjrab National Park Gilgit, Pakistan	2011	43	28	6	13.5	86.5	112	0.67	Khan et al., 2011 [81]
7	Khushab, Pakistan	2011	48	32	26	54.5	45.5	92	3.56	Qureshi et al., 2011 [99]
8	Hingol National Park Baluchistan, Pakistan	2012	39	22	10	25	75	102	1.35	Qureshi, 2012 [100]
9	New Murree, Patriata, District Rawalpindi	2013	93	56	14	30	70	90	1.69	Ahmed et al., 2013 [22]
10	Karak, KPK	2014	160	50	50	68.2	31.8	67	6.32	Khan et al., 2014 [48]
11	Tehsil Kabal, Swat, KPK	2015	45	27	19	42.2	57.8	99	2.68	Ahmad et al., 2015 [21]
12	Tehsil Chakwal	2009	29	18	12	34	66	97	1.67	Qureshi et al., 2009 [29]
13	Tehsil Kharian, District, Gujrat	2014	50	32	27	51.5	49.5	93	3.47	Ajaib et al., 2014 [106]
14	Ladha Sub Division, South Waziristan agency, Pakistan	2016	82	42	13	30.4	69.6	93	1.78	Aziz et al., 2016 [81]
15	Bhimber, Azad Jamu Kashmir	2011	38	22	12	34	66	95	1.67	Mahmood et al., 2011 [107]
16	Himalayas Mountain Naran Valley	2013	101	52	40	61	39	112	5.87	Khan et al., 2013 [57]
17	District Mirpur AJK, Pakistan	2011	29	20	14	30	70	102	1.69	Mahmood et al., 2011 [89]
18	District Gujrat	2013	22	18	7	31.8	68.2	111	1.98	Parvaiz, 2014 [90]
19	District Sialkot	2014	18	13	11	27.7	72.3	113	1.57	Ikram et al., 2014 [100]
20	Valley Alladand Dehri, Tehsil Baathkhela, District Malakand	2013	92	53	45	74	26	94	6.14	Alamgeer et al., 2013 [85]
21	District Swabi, Pakistan	2017	66	41	7	22.7	77.3	103	1.34	Rozina et al., 2017 [108]
22	District Kotli, Azad Jamu Kashmir, Pakistan	2010	38	25	4	13.1	86.9	113	0.56	Ajaib et al., 2010 [109]
23	Mianwali District	2007	21	16	8	61.9	38.1	105	0.68	Qureshi et al., 2007 [27]
24	Tehsil Dargai, District Malakand	2013	40	26	23	22.5	77.5	109	3.35	Zaman et al., 2013 [87]
25	Sudhan Gali and Ganga Chotti Hills, District Bagh, Azad Kashmir	2007	33	17	3	3.03	96.6	117	0.34	Qureshi et al., 2007 [67]
26	Hattar Region, District Haripur, NWFP	2008	45	26	25	55	45	89	3.45	Hussain et al., 2008 [50]
27	Tehsil Kotli Sattian, Soan River, Rawalpindi	2016	35	20	13	37.14	62.85	105	2.31	Bashir and Ahmad, 2016 [110]
28	District Kotli Azad Jamu Kashmir	2014	93	46	38	27.96	72.05	92	3.98	Ajaib et al., 2014 [111]
29	Neelum Valley, AJK, Pakistan	2011	40	31	5	12.5	87.5	113	0.59	Mahmood et al., 2011 [112]
30	Vehari, Pak Pattan, Lahore, Faisalabad, Nankana Sahib, Sahiwal, Sialkot, Narowal and Central Punjab	2013	51	5	40	44	60	111	6.12	Zereen, 2008 [88]
31	Eight Districts of Punjab, Vehari, Pak Pattan, Lahore, Faisalabad, Nankana Sahib, Sahiwal, Sialkot, Narowal	2012	48	23	16	33.33	66.66	102	2.45	Zereen et al., 2013 [113]
32	Field survey of the Punjab	2012	36	13	9	13.88	86.11	113	0.79	Iltaf et al., 2012 [114]
33	Erer valley of Babile Wereda Eastern Ethiopia	2012	51	28	4	7.84	92.15	114	0.35	Belayneh et al., 2012 [68]
34	D.I. Khan, Bannu, Lakki Marwat, Karak and Kohat KPK	2015	52	36	13	36.5	63.4	99	2.34	Tariq et al., 2015 [115]
35	Indus River, dera Ismail Khan, Pakistan	2014	70	39	13	37.14	62.85	92	2.34	Mussarat et al., 2014 [94]
36	Western Uganda	2014	231	72	50	0.86	99.13	116	6.93	Asiimwe et al., 2014 [66]
37	Manila Philippines	2017	76	40	12	6.57	93.42	113	2.18	Lloyd et al., 2017 [116]
38	Susunia hill of Bankura District, West Bengal, India	2015	25	17	9	20	80	113	0.79	Rahaman and Karmakar, 2015 [117]
39	Kalenga Forest Area Bangladesh	2014	35	25	18	17.1	82.85	112	2.88	Uddin and Hassan, 2014 [118]
40	Samburu Community Wamba, Kenya	2009	33	5	6	3	97	117	0.45	Omwenga et al., 2009 [69]
41	Samahni, District Bhimber Azad Jammu and Kashmir, Pakistan	2021	150	58	42	40	60	85	4.26	Ishtiaq et al., 2021 [118]
42	Chenab riverine area, Punjab province, Pakistan.	2019	129	59	57	48	52	95	5.25	Umair et al., 2019 [119]
43	flora of Gujranwala region, Punjab, Pakistan	2020	100	52	43	45	55	80	4.23	Iqbal et al., 2020 [120]
44	Jhelum District, Punjab, Pakistan	2021	57		22	35	65	77	3.25	Majeed et al., 2021 [121]
45	Harigal, Azad Jammu Kashmir.	2021	150	60	29	25	75	60	2.95	Amjad et al., 2021 [122]
46	Gokhand valley, KPK.	2020	109	64	30	32	68	90	3.47	Sulaiman et al., 2020 [123]

#### Comparison with other studies of adjacent areas

Only a few researchers developed formulations and recipes and they are confined to only a few plant species. Because traditional knowledge about wild plant resources spread in such a unique way that this industry attracted a specific type of person. In recent decades, it has been found that a lack of interest among young has resulted in a knowledge transformation gap, highlighting the importance of ethnomedicinal studies. West Pakistan produced the first document relating to 1,500 therapeutic plant species [70, 71].

It is worth noting that different plant species are utilised to cure a variety of diseasees. One plant species can be used alone, in combination with other plants, or in a blend of diverse compounds to cure various diseases. Therefore, various plant recipes were used to cure ailments in typical areas. Interestingly it was also observed that some of the plants have specific application while others have multiple uses like *Cassia fistula* and *Tamarindus indica*. One teaspoon amaltas fruit pulp and an equal amount of tamarind in one cup of water, left overnight mashed and strained is used for stomach problem.

Similarly, one plant species can be used to treat many diseases, such as *Amaranthus spinosus*, which is used as an antidote and for constipation. In addition, a single ailment, such as asthma, can be treated using a wide range of plant species. Medicinal and industrial uses may be found in many wild plant species. *Eucalyptus globulus* is used as a culinary ingredient, a component of pharmaceutical formulations, and in the manufacture of furniture and sporting products. The results of this study indicated that *Saccharum spontaneum* L., a member of the poaceae family, was one of the earliest species to be investigated for different therapeutic applications, including constipation, burning sensation, phthisis (pulmonary TB), and blood disorders.

In Pakistan, India, Nepal, Iran, Morocco, Singapore, or Kenya, this species’ medicinal applications have never been documented [72–78]. Eight leguminosae species have been recorded from diverse sites on Head Maralla. This family is well-known in the pharmaceutical and food sectors, and they work with both people and animals. Members of this family include a lot of phytochemicals such tannins, phenol, alkaloids, conmarins, glycosides, lignin, quinones, and steroids. In addition to ethnomedicinal properties, it is a source of protein, wood, fibre, gums, resins, colouring matter, insecticides, and molluscicides [79, 80]. Fodder species of this family are used to treat many diseases in livestock. Current study might lead to the formation of a new drug. They might also be utilised to find active phytochemicals that could be used instead of medicines. The study conducted in Khunjerab National Park, Gilgit Pakistan, and Ladha subdivision, South Waziristan Agency, Pakistan, reported that many species of this family are utilized for milk production, skin infection and lung diseases in animals [81, 82].

*Malva sylvestris* L. (Khabzi), *Malva parviflora* L. (Sonchal), and *Bombax ceiba* L. (Sumbal) are members of the Malvaceae family. Tannins, polysaccharides, coumarins, flavonoids, malvin, folic acid, terpenoids, vitamin A, vitamin C, and vitamin E are among the phytochemicals found in this family [83]. Because of these phytochemicals, they can be used to treat a variety of human and animal diseases. These species are used to treat kidney problems, sex organs, viral infections and bacterial diseases. Tree bark has been reported to have high medicinal values in the finding from current study [84]. There is a need to examine it further for active pharmacological components. Skin illnesses, fodder, ornamental, stomach problems, demulcent, smallpox, malaria, TB, renal diseases, allergies, athlets’ foot, and ringworm are all treated with *Artemisia scoparia*, *Xanthium stromarium*, *Eclipta alba*, *Eclipta prostrata*, and *Carthemus oxycantha* (family Compositae). It may also be used as an air tonic and to treat bleeding issues, jaundice, fever, toothaches, and ulcers. This family contains active compounds [85].

This means that target family members are being employed to treat both human and animal illnesses. Only one research documented the applications of *Carthamus oxyacantha* M. Bieb., which included using its leaves in modest quantities to treat intermittent fever, wounds, ulcers, and chornic sores, and applying a poultice of gently roasted leaves to decrease inflammatory swellings and rheumatism. Fermented leaves reduce chest discomfort and heal tympanitis, while recent research has shown novel uses for seed oil, such as treating ulcers, toothaches, and itch. As a result, new sources of medicine might be investigated for the preparation of novel medications, either alone or in combination [86].

*Mentha spicata* (podina), *Mentha longifolia*, and *Leucas aspera* are commonly grown species in the Lamiaceae family and used in digestive/gastric problems, asthma, jaundice, chronic diseasees, as well as salad and fodder. This family is well knownfor many well know plant products and chemical compounds [87]. These species have been known to be used as a part of local culture for millennia. Fresh leaves have been shown to be edible and might be utilised as a carminative for diarrhoea, dysentery, and colics in previous research [88]. Whereas recent research is the first report from Head Maralla on novel applications of *Leucas aspera* (Willd.) Link in asthma, jaundice, and chronic diseases. The current study provides a foundation for determining the biological activities of these important plants in order to create novel antiseptic and insecticidal drugs [89]. *Chrozophora tinctoria* (family Euphorbiaceae) was used for wound healing at Head Maralla, although it was also used for jaundice, typhoid, vomiting from seeds, and the plant yields colouring matter in the literature [90]. It was also utilised as a stomachic for chest burning in another research [91]. *Artemisia scoparia* is used for skin disorders, as fodder, and as a decorative, and it is diuretic in nature [36], but it has also been recorded for earache, heart problems, fever, and blood pressure [84, 92, 93]. Diarrhea, bleeding, and haemorrhoids were all treated by *Erigeron bonariensis*. Additionally, the leaves were utilised to cure diarrhoea and diabetes. In the Navapind and Shahpur Virkan areas, it is said to be used to treat asthma and ulcers [36]. It has been used for bleeding and as a diuretic in the literature [6, 84, 94]. E. prostrata was discovered to be effective in the treatment of allergies, athlete’s foot, and ringworm. It’s also utilised for urticarial and blood purification. It has been reported in the literature to be used as a scorpion antidote and for constipation [36, 95].

*Parthenium hysterophorus* is used to treat skin disorders and is frequently used internally to treat a variety of ailments. Previous research has discovered that it can be used to treat blood purification, backache, diarrhoea, fever, and toothache. [36, 96–99]. Another plant species, *S*. *marianum*, was utilised to treat liver problems, chronic inflammatory conditions, and heartburn. Furthermore, it has been shown to be helpful against cancer, wound healing, and TB [36, 45]. *E*. *helioscopia*, a member of the Euphorbiaceae family, was used for eruption and cholera therapy, but it was also described as being used for cancer and cholera treatment in a research by Shahpur Virkan and Navapind [36].

*Ficus religiosa* was used locally to treat constipation, vomiting, asthma, and urinary issues, and it has also been used in the literature to treat constipation, wound healing, diarrhoea, ulcer, molar pain, and cardiac disorders [36, 100–102]. *Ficus benghalensis* is reported to be used for sex power and jaundice, while earlier research has suggested that it might be useful for diarrhoea, blood purification, and diabetes [36, 103, 104].

Another significant plant, *Portulaca oleracea* was discovered during the current research. This was used to treat kidney infections, painful urination, jaundice, iron deficiency, and skin allergies among the locals. Previously, it was only found to be beneficial in the treatment of urinary and intestinal disorders in trials. Juice’s diuretic action makes it beneficial in the treatment of bladder problems. The mucilaginous characteristics of the plant also make it a calming treatment for gastrointestinal issues including dysentery and diarrhoea. These studies support current results that seeds are emollient, water pilling, and effective for internal worms [105]. *Digeria arvensis* Forssk was discovered to be useful for headaches, burning, dyspepsia, urination, and constipation. It is also used as a salad, vegetable, and fodder. In Khushab regions, the leaves of Digeria arvensis was employed as a potherb for curing constipation [106]. It’s worth noting that the climate in Head Maralla differs from that of Khushab, which is more or less arid and semi-arid. As a result, the locals employed these plants to meet a variety of requirements.

New usage discoveries may open novel avenues for phytochemists, pharmacologists, and even local herbalists in developing new medications and reaping the benefits of nature’s health resource. Similarly, the matured fruit of Cucumis melo was consumed and described as moderate constipation in Hingol National Park, Baluchistan, Pakistan [107]. Current research, on the other hand, indicates that *C*. *melo* was utilised as a tonic and as animal feed in the Head Maralla area. This report might lead to the discovery of a new supply of feed.

According to published data, Adiantum capillus-veneris is used to treat a variety of diseasees, including colds, coughs, flues, and asthma [39]. Recent investigations have revealed that it was utilised for bronchial disorders in the Head Maralla region. It’s also the first time this plant species has been used in a novel way. Furthermore, new findings have been made on the pharmacological characteristics of *Convolvulus arvensis* L., which have been utilised in the Head Maralla region for fever wound healing, and menses. The local communities of high altitude area of Himalayan region also used *Convolvulus arvensis* L. in the form of powder which is purgative & effective in bowels [39]. This plant should be investigated further in order to discover novel phytochemicals that might lead to the creation of new medicines. Earlier studies from the Sialkot area indicated that *Eichhornia crassipes* was utilised in skin treatments and to treat goitre, but new research from Head Maralla discovered it as a multifunctional plant that may be used as an antioxidant, a carotene source, and as manure [108]. As a result, it is recommended that its traditional wisdom be assessed not only from a medicinal standpoint, but also as a source of supplemental food and natural manure for vegetables and agricultural plants.

#### Recipes used in Head Maralla area

Local people used a variety of recipes for their day-to-day need (Table 2). For stomach and digestive problems, leaf powder of *Mentha spicata* L. and their extract should be taken two to three times orally. Crushed leaves are also used as a ‘chatni’ (sauce) for eating, aiding digestion and providing a fragrance derived from tiny mentha bits. Chatni is a cooling and digestive drink that also contains chunks of unripe mango fruit to enhance flavour. Boiling the leaves of Mentha longifolia L. has been shown to be beneficial in decreasing mouth odour.

*Melia azedarach* (Dherak) fruit/seeds were also crushed and used to reduce edoema from bowls. The paste made from the leaves is often used to treat skin problems. Another typical method for this plant is to boil entire leaves for half an hour and then wrap in a piece of fabric, which may be used to treat wounds and remove the symptoms of bug bites. Crushed seed extract was also used as a tonic to treat pimples and other long-term skin diseasees and disorders in rare situations. *Chenopodium album* L. (bathu) is used to create saag, a vegetable similar to *Brassica campestris*. Crushed leaves are combined with palak (spinch) and spices, then cooked for an hour and a half to produce a paste that resembles vegetable cabbage.

Another wild plant *Achyranthes aspera* is effective for joint pain by making paste of the roots and soaking it for four to five hours. Itching and skin infections can also be treated with root paste and boiling extract. *Scandix pectin-veneris* L. leaves and blossoms were used as a salad and vegetable. *Eclipta prostrata* leaf extract was also utilised as a hair tonic, resulting in glossy, dark, and healthy hair. It also aids in the reduction of baldness and the rejuvenation of hairs.

This discovery might lead to the development of novel cosmetics. *Chenopodium murale* (Krund) was another valuable plant, as the entire plant may be utilised as an insect/pest repellant. Leaves may usually be stored in grain storage areas. *Euphorbia helioscopia* L. (gundi buti) latex was applied to eruptions, and seeds with pepper were administered to cholera patients. Furthermore, *Euphorbia prostrata* Aiton paste was used in conjunction with lemon extract to treat skin disorders, itching, and ringworms on the body. Plants from the *Alhagi maurorum* genus are frequently used to treat skin allerigies and teeth cleaning. Seeds of *Albizia lebbeck* (L.) Benth have been orally proven useful were used to eat orally and proved effective against many diseases.

According to literature, another species was *Ipomoea carnea* Jacq., which was used to treat jaundice. Its seeds are combined with honey and castor oil to cure worms and intestinal discomfort. Swelling was treated with seeds and vinegar. Recent research has shown that this plant is anti-carcinogenic and oxytoxic properties, and it is used treat asthma, insect bites, and burns [7].

*Cichorium intybus* L. also has a variety of advantages when employed in various dishes, such as when the leaves were eaten as a vegetable. As a coffee adulterant, the roasted root was employed. The root and leaves were used as an appetiser, a depurative, a digestive, a diuretic, a constipation treatment, and a tonic. The latex in the stems was applied on warts to kill them, and a decoction of the freshly picked plant was used to cure gravel. Blood glucose levels can also be regulated by taking *Cichorium intybus* L powder twice a day. Similarly, chewing 4 to 5 leaves of *Zizypus jujube* Mill. on regular basis help to regulate blood glucose levels. Furthermore, a teaspoon of *Melia azedarach* L. powder was found to be beneficial against diabetes when taken daily before breakfast for a month.

In addition, the latex of *Ficus bengalensis* L. leaves and branches, when combined with honey and taken orally, can help with diabetes. Another usage of *Justicia adhatoda* L. was to treat respiratory infections with its leaves, which contain the alkaloid vasicine, which has significant bronchodilator action and may be taken as a juice or decoction. Leaves are used topically as a poultice to heal wounds and joint discomfort because they have antibacterial and anti-inflammatory qualities. Syrup made from *Justicia adhatoda*, help expectoration, relieves bronchial spasms, and restores normal respiratory function. Menthol, which is derived from Mentha, has been utilised in a variety of medicines. Breathing becomes more refreshing as a result of it. *Morus nigra* L. extract was used to make the popular ‘Sharbat tootseha’ syrup, which is beneficial against throat infections and discomfort. It can also help to increase the size of the glands in the neck. Three to four times a day, ten millilitres, or roughly two teaspoons, can be utilised to generate beneficial results. Fresh aerial portions of the plant *Solanum nigrum* L. are used as a vegetable in cooking and are used for diabetes control. Aqueous extract of the *Oxalis corniculata* L. plant was used as a drink and cooling agent for stomach problems. The leaves’ extract was used to alleviate discomfort and reduce swelling and redness in the eyes. To stop bleeding from a wound, a paste made from fresh leaves was applied. These recipes have a lot of potential to be evaluated scientifically before being translated into medicinal goods.

### Uniqueness/novelty of the findings and future prospectus

The research area is located at the union of three rivers (Jammu Tavi, Manawar wala Tavi, and Chenab River), all of which provide very fertile soil as well as water flow, making it ideal for a variety of flora. The majority of the vegetation was unique to each location (Table 2 and Figs 1 and 2). Site 1 was dominated by *Justicia adhatoda* L., *Lantana camara* L., site 2 was dominated by *Canabis sativa* L., *Sonchus asper* (L.) Hill, at site 3, *Fumaria indica* (Hausskn.), *Solanum xanthocarpum* Schrad. & H. Wendl., *Typha latifolia* L., were present. Unique plants at site 4 were as *Dalbergia sissoo* DC., *Ficus benghalensis* L., and *Acacia modesta* Wall.

Furthermore, certain bryophytes and fern species were unique to the studied region. *Marsilea quadrifolia* (aquatic fern), *Osmunda regalis* L., *Marchantia polymorpha* L., and *Riccia cavernosa* Hoffm. *Azolla pinnata* R. Br., *Marsilea quadrifolia* (aquatic fern), *Osmunda regalis* L., *Marchantia polymorpha* L., and *Riccia cavernosa* Hoffm. Furthermore, *Spirogyra buchetii* Petit was present throughout the season, but *Chara Schweinitzii* A. Braun. was only present in the fall. Previously, study conducted by Tariq et al. [114] has been focused on the documentation of diversity in Punjab and neighboring areas of Azad Kashmir and less attention was paid on medicinal importance of native plants of the area. However, recent research has revealed the economic significance of certain plants, such as *Azolla pinnata*, which is utilised as a green manure in rice fields to provide nitrogen and organic matter to the soil. It also has the ability to phyto-remediate contaminants in the environment. This could further lead to develop new form of fertilizers or compost making. Likewise, *Osmunda regalis* is used medicinally for blood purification and to treat renal diseases. The roots of same plant are used for the production of fibre and whole plant is eaten as food.

## Conclusion

The findings of this study certainly open new avenues for research and development. Focus on particular flora shall resultantly bring a systematic approach to cultivate and harvest unique ideas and fruitful outcomes. There is dire need to expand the collection, exploration mission and documentation of the particular flora because in this area seasonal streams and nullahs are flowing which support unique plants to grow in different seasons. It is assumed that efforts involving the native people and other stackholders from different governamental departments for new plantation, cultivation, harvesting, and post-harvesting will have the greatest impact on overall vegetation of the area. The Head Maralla is a hub of unique plant variety, wildlife, and bird fauna. Conservation efforts with the involment of local community, university faculty and students, local government, irrigation department, forest department, tehsil municipal administration, and civil servants for new plantation, cultivation, harvesting and post harvesting will result in higher benefits. The studied area should be classified as a protected wetland under the Convention on Wetlands Conservation. The area needs concentrated and coordinated efforts to protect the native flora. Plant biologists and forest service officials have numerous opportunities to collaborate and expand plantation across both districts and rivers through motivation and support. This document would be a scientific contribution towards preserving traditional knowledge of wild plants of the area and foundation for future conservation efforts.

## Supporting information

S1 File (DOCX)

## Abbreviations

TRM: Traditional medicines
PHC: Public Health Committee
